RETRACTED

# Changes in the Surface Water Nitrogen Content in the Upper Hun River Basin, Northeast China

**DOI:** 10.1155/2022/4175218

**Published:** 2022-07-31

**Authors:** Wenkai Jin, Jian Ma, Xin Chen, Guohui Yan

**Affiliations:** ^1^Key Laboratory of Pollution Ecology and Environmental Engineering, Shenyang Institute of Applied Ecology, Chinese Academy of Sciences, Shenyang 110016, China; ^2^University of Chinese Academy of Sciences, Beijing 100049, China; ^3^Binzhou Business Environment Construction Service Center, Binzhou 256600, China

## Abstract

Human activities have considerably increased nitrogen intake into waterways, resulting in the deterioration of water quality. The state of surface water requires special consideration in light of the water crisis caused by nitrogen pollution. In this study, the natural abundance of the nitrogen stable isotope (*δ*^15^N) is measured and sampled in sediments and compared with the total dissolved nitrogen (DN) in four main Chinese tributaries of Hun River upper reach, including the Dasuhe, Beisanjia, Beikouqian, and Nanzamu tributaries. Results show that for the Dasuhe and Nankouqian tributaries, the *δ*^15^N values of sediment samples in 2016 are all significantly higher than previous values in 2011. In the Dasuhe tributary, this change is attributed to the promotion of organic agricultural production under which chemical fertilizers are replaced by organic fertilizers. For the *δ*^15^N values of the sediment in the Nankouqian tributary, the construction of the municipal sewer system and wastewater treatment facilities are the causes of this rising trend. The *δ*^15^N values of nitrate released by facilities could be raised by microbial denitrification that is employed in the tertiary treatment process. Most of the *δ*^15^N values of the sediments are distributed between soil and manure, indicating that nitrogen in the river water mainly comes from agriculture. All the surveyed tributaries except Dasuhe show a significant increase in DN. In addition, a significant positive correlation between the change ratio of the farmland area and DN in river water is observed, suggesting that the increase in nitrogen in river water from 2011 to 2016 is due to agriculture. Based on the abovementioned data, this study provides a basis for local governments to formulate management measures.

## 1. Introduction

Nitrogen (N) is a vital nutrient for ecosystem function and a limiting component in the productivity of many ecosystems across the world [1]. Nitrogen pollution can have negative ecological impacts, such as soil acidification, hypoxia, and eventual fish death [2]. Eutrophication of the aquatic environment is caused by high nitrogen concentrations, which result in a loss of biodiversity and worsening of the water quality [3]. To make matters worse, elevated nitrogen levels in drinking water have been linked to an increased risk of human illness [4]. How to make rational use of nitrogen and reduce its negative effects of nitrogen while meeting human needs has become a scientific challenge that human beings must solve in the 21st century [5].

RETRACTED

The excessive application of artificial nitrogen (N) is posing a threat to human health and the earth's ecological balance [3, 4]. To resolve these problems, efforts around the world are underway to reduce nitrogen input to water source areas by changing land-use patterns [6], building wastewater plants [6], or improving agriculture practices [7]. Most environmental management systems in China have committed to improving urban and industrial environments during the last 20 years [8]. However, agriculture is responsible for more than half of the excess nitrogen entering waterways worldwide [9]. The vulnerability of the aquatic ecosystem is increased by land use/cover change (such as farming expansion, afforestation, deforestation, urbanization, and industrialization), which is a key manner and reaction of human activities to the surface environment [10]. Sewage is the primary source of nitrogen in industries, cities, and people's lives. Fertilizers, nitrogen-fixing crops, human and animal excreta, and soil erosion induced by land-use changes such as deforestation and grassland restoration are all examples of agricultural nitrogen fertilizers. Construction sites give nitrogen to water bodies as well [11]. Land use in settlement areas, particularly in agriculture, has a significant impact on nitrogen levels in surface water [12]. Zhao and Huang [12] discovered that when forest proportion increased, nitrate levels declined. Water yield is increased when a paddy field is converted to dry ground or construction land, whereas water yield is reduced when a water area is converted to a paddy field or dry land. Based on a geographic information system (GIS) spatial analysis employing land use covers, Yuxian et al. [13] investigated the geographical link between anthropogenic activity and water nitrogen on the eastern Loess Plateau. On the Watershed Scale, three human land use categories and two nitrogen indexes were employed to assess the rivers' condition. The findings revealed that river nitrogen levels were directly linked to human land use patterns. In metropolitan areas, nitrogen pollution was the worst. The authors in [14] reported that forest and agricultural cover types play important roles in predicting the surface water quality during the low-flow, high-flow, and mean-flow periods.

RETRACTED

Since the 1990s, the water quality of the Dahuofang reservoir (DHF), which generates drinking water for 23 million people [15], has gradually deteriorated, mainly due to excessive nitrogen emissions [16]. To avoid further decline in the water quality to a level that threatens human health, a series of Chinese government measures have been implemented to reduce nitrogen content in the Upper Hun River (HR) Basin, which is the main watershed area of the DHF [14]. Since 2014, 2,513 ha of farmland around the main watershed area of the DHF have been returned to forest or grassland and are mainly distributed across the Dasuhe, Nankouqian, and Nanzamu tributaries. In addition, Qingyuan County, which is in the upper reach of the Hun River watershed, has upgraded three major wastewater treatment facilities (WTFs) that directly discharge into rivers. Together, many sewage treatment facilities in villages and towns were built between 2014 and 2015 [17].

The natural abundance of the nitrogen stable isotope (*δ*^15^N) is a reliable indicator in tracking anthropogenic nitrogen inputs to aquatic systems [18]. In river systems, water, sediment [19], and biota *δ*^15^N values change with the N source [20]. This distinct feature makes *δ*^15^N a signature among N sources in the intensive cropping and livestock farming system. Moreover, in sewage treatment facilities or groundwater influenced by septic systems, nitrogen has elevated levels of ^15^N relative to ^14^N [21]. Sediment is less disturbed and can reflect long-term accumulation [22]. Therefore, monitoring changes in *δ*^15^N over time at specific locations could reveal the sources and reflect the variety of nitrogen input into rivers.

In this study, nitrogen isotopes are collected from sediments of four main tributaries of Hun River upper reach, including Dasuhe, Beisanjia, Nankouqian, and Nanzamu. The isotopes are sampled and assessed to measure the change in agricultural and sewage management measures from 2011 to 2016. A significant positive correlation between the change ratio of farmland area and DN in river water is observed, suggesting that the increase in nitrogen in river water from 2011 to 2016 is due to agriculture.

The rest of the manuscript is organized as follows: Section 2 is about material and methods and provides a detailed description of the data collection, sampling, and analysis.  Section 3 illustrates different results for nitrogen concentration and Section 4 is about the discussion. The conclusion is presented in Section 5.

## 2. Materials and Methods

### 2.1. Research Area

The details on the changes in background information from 2011 to 2016, including population density and farmland area percentage, for the four tributaries' including Dasuhe, Beisanjia, Beikouqian, and Nanzamu are listed in Table 1.

RETRACTED

### 2.2. Sampling

In this study, the sampling time was set in September to reduce the impact of rainfall. Sediment and water were collected from every 24 stations in the upper reach of the Hun River watershed, Northeast China. These sampling locations included four chief tributaries that are locally classified as upper (Dasuhe), middle (Beisanjia and Nankouqian), and lower (Nanzhamu) portions of the Upper Hun river watershed. Six sampling locations were added in this investigation that were distributed along the mainstream of the Hun River from east to west. Information on the sampling locations and the WTF running status in this area during this investigation are presented in Figure 1.

The sediment thickness at most sampling sites is relatively shallow (<5 cm), while some are thicker. Under these circumstances, the sediment was sampled with the greatest depth of 5 cm. Moreover, soil, chemical fertilizers, livestock manure, and wastewater samples in this area were also collected to determine *δ*^15^N values of common nitrogen sources in rivers in this area. The details are listed in Table 2. Solid samples were sampled and sealed in disposable plastic automatic sealing bags, while water samples from each site were stored in polyethylene plastic bottles prerinsed with distilled water. All the samples were kept below 4°C and transported to the laboratory for further analysis.

### 2.3. Sample Preparation and Isotopic Analysis

Solid samples were placed in aluminum pans which were dried at 60°C for 24 hours. Dried samples were then ground to a fine powder with a mortar and pestle until they could all pass through a sieve with a diameter of 0.15 mm. The ground samples were stored in glass vials until analyzed. About 50 mg of each solid sample was weighed into a tin boat and analyzed for N isotope and total nitrogen (TN) using a Finnigan MAT DELTA plus XP stable isotope ratio mass spectrometer. A urea nitrogen isotope standard (*δ*^15^N = −0.45%) was used to determine against the instrument every 10 samples. The average isotopic difference measured for these standards was less than ±0.15% for *δ*^15^N and ±0.01% for TN values. Water samples were filtered using Millipore filters (0.45-*μ*m pore size, MF-Millipore) before analysis. Dissolved inorganic nitrogen (DIN), including NH_4_^+^, NO_2_^−^, and NO_3_^−^ was measured by ion chromatography DIONEX ICS-900, while dissolved nitrogen (DN), including both organic and inorganic N in the water-soluble form, was analyzed by using an Analytik-Jena multi N/C® 3100 analyzer.

RETRACTED

### 2.4. Statistical Analyses

Statistical regression was used to test the relationship between water DN and sediment TN at each sampling location. No significant relationships were observed in both the two sampling periods. Dissolved nitrogen at each location was also not significantly correlated to sediment *δ*^15^N. A two-factor analysis of variance (ANOVA) was used to make *δ*^15^N values statistical analysis, with sampling year and tributaries being the main factors. For each analysis, overall F-tests with an alpha <0.05 were used. All statistical analyses were performed on IBM SPSS Statistic software version 21.0 [23, 24].

## 3. Results

### 3.1. Water Nitrogen Consistency Change

A different general trend of water DN was observed when comparing site values from the source to the outlet at each tributary in the two sampling periods. In 2011, except for the tributary around the DHF, the DN values in most tributaries showed a downward trend from the source. In contrast, no simple trend could be used to profile the changes in DN values down the river for the four tributaries in 2016. However, in the three tributaries west of Dasuhe, the mean DN values of each tributary were higher than those in 2011. The results are shown in Figure 2. Similarly, the mean DIN to DN rates in more eastern tributaries, including Dasuhe and Beisanjia, were higher than the data in 2011, while the other two western tributaries showed a reverse trend (Figure 2). In the Hun River mainstream, inorganic nitrogen values were generally around the value of 3 mg/L. As shown in Table 3, the dissolved nitrogen in this river extensively varied and did not show a clear trend from the source to the DHF in 2016.

Compared to the mean values of DN, those of Nankouqian and Nanzamu were higher than those of the mainstream, while the other two were lower.

### 3.2. Sediment TN and Nitrogen Isotope Change in Tributaries

For the tributaries near the source of the Hun River, including Dasuhe and Nankouqian, the same general trend was observed for the 2016 sampling period as previously reported in 2011. The details are shown in Figure 3. In these tributaries, the sediment *δ*^15^N values generally increased from the source of each river to the sampling locations near the tributaries' outlets. However, a downstream decreasing trend in *δ*^15^N for Beisanjia and slight variability for Nanzamu show that the two tributaries were different in 2011. In 2011, the mean *δ*^15^N values of each tributary were Nanzamu > Beisanjian > Nankouqian > Dashuhe. However, in 2011, the pattern was Nankouqian > Nanzamu > Dashuhe > Beisanjia. Despite no significant differences between the four tributaries in each sampling year (*P* > 0.05, *F* = 2.547 in 2011, *P* > 0.05, *F* = 1.129 in 2016, 3 degrees of freedom (d*f*) per contrast), the *δ*^15^N values were significantly different in the two sampling periods (*P* < 0.05, *F* = 10.992 1 d*f*). Except for the three sites in the Bersanjia and Nanzamu tributaries, the *δ*^15^N values for sediment samples collected during 2016 were generally higher than those in 2011.

RETRACTED

For the Bersanjia and Nanzamu tributaries, no clear trends between the sampling years 2011 and 2016 were observed for each site. However, for Dasuhe and Nankouqian, the sediment samples *δ*^15^N values were all significantly higher than previous values. These rises in *δ*^15^N generally ranged from 0.8% to 3.4% for the two tributaries (Dasuhe, *P* < 0.01, *F* = 87.76; Nankouqian *vs*. *P* < 0.01, *F* = 25.58 1 d*f*).

Figure 4 shows that the mean sediment *δ*^15^N values in the four tributaries all increased in 2016 than those sampled in 2011. No significant relationships between the 2016 human population density of the watersheds and the percentages of villages (rate of villages to the whole sub-watershed area) were observed as previously reported. The outlet *δ*^15^N data of each tributary also showed the same correlation.  Figure 5 shows the range of the sediment *δ*^15^N value and TN concentration in each sampling point. For the relationship of sediment *δ*^15^N values versus TN concentration, most sediment *δ*^15^N values of tributaries were between the range of soil and livestock manure in this area (Table 2).

### 3.3. Sediment Nitrogen Isotope Trend in Hun River Main Stream

Sediment *δ*^15^N values in the mainstream covered the range of soil to livestock manure (Table 3 and Figure 5) and showed a trend that is more steady with the distribution of WTFs (Figure 1). The mainstream mean nitrogen isotope value was (*δ*^15^N mean value: 7.6%) significantly higher than the other three tributaries collected in 2016 (*δ*^15^N mean values: Dasuhe, 5.6%, *F* = 16.2; Beisanjia, 5.1%, *F* = 14.1; Nanzamu, 6.3% *F* = 8.5, *P* < 0.01 for all pairs). The exception to this was the Nankouqian tributary, which showed a *δ*^15^N mean value of 7.7%.

### 3.4. Correlation Analysis of the Change Rate of Total Nitrogen Dissolved in River Water and Change Rate of Farmland Proportion

Although farmland area percentage and population density are not related to DN in the entire basin, a significant positive correlation was found between the change in the ratio of farmland area and mean DN in the river water (Figure 6). It explained that the increase in nitrogen in the river water from 2011 to 2016 originated from agriculture. Hence, we inferred that organic fertilizers were excessively used.

RETRACTED

Farmers are not aware of the dangers of excessive nitrogen emissions to humans, and only sewage and garbage are classified as pollutants. In the practice of replacing chemical fertilizers with organic fertilizers, too much organic fertilizer was applied just in case of production reduction. Even in a few fields, chemical fertilizers are still secretly applied.

## 4. Discussion

Dasuhe and Nankouqian tributaries showed the most extensive increase in sediment *δ*^15^N values during the two sampling periods. In Dasuhe, this change may be due to the chemical fertilizer replacing action (government documents). Since 2014, the local government has encouraged farmers to use organic fertilizers made from livestock manure from local poultry and pig farms to replace chemical fertilizers to reduce nitrogen input to rivers by external chemical fertilizers. These actions may have contributed to the changes observed in this river system as the sediment *δ*^15^N values were mainly in the range of soil and livestock manure (Table 2), which was much higher than chemical fertilizers collected in this area. In terms of the *δ*^15^N change in the Nankouqian tributary, the construction of the municipal sewer system and wastewater treatment facilities may account for this increasing trend. Many residences in municipalities along the Nankouqian tributary have been linked to the municipal sewer system since 2012, whereas undeveloped villages have open drains with oxidation ponds. The *δ*^15^N of the nitrate released by facilities could be increased by microbial denitrification that is employed in the tertiary treatment process [25]. However, the intermittent running state of WTFs in this tributary could be one of the reasons why dissolved nitrogen values in rivers were higher than those in 2011. Except for sites HR9 and HR10 which are located downstream of WTF (Figure 1), most *δ*^15^N values of the sediments were distributed between soil and manure (Figure 5), indicating that nitrogen in river water mainly comes from agriculture.

No significant change in DN was observed in the Dasuhe Tributary. This is mainly due to the minimum farmland area percentage and a large area of primary secondary forest, making the effect of human events drop to the lowest. For the other three tributaries, DN in river water significantly increased. Since there was no significant change in the annual rainfall on record between 2011 and 2016 according to the local weather bureau; the reason for the increase in DN may be an increase in the amount of nitrogen discharged into the river water [26, 27].

The local Environmental Protection Agency lacks long-term monitoring of water quality in tributaries. Most fixed-point monitoring points are concentrated around the DHF reservoir, resulting in the lack of basic data on the sources of river water nitrogen. It is thus almost impossible for researchers to continuously monitor such vast waters. As daily necessities become more abundant in rural areas, the range of nitrogen stable isotopes from domestic wastewater is larger than before. Using only stable isotope technology to analyze nitrogen sources may thus not be accurate. Something more stable and more relevant to life such as plasticizers could be used together with a stable nitrogen isotope to identify nitrogen from domestic wastewater [28, 29]. Also, during the research, we found that the organic nitrogen content in the water is complex, and determining the composition of organic nitrogen would be one of the next research directions.

RETRACTED

## 5. Conclusions

Nitrogen pollution has several negative ecological impacts, including soil acidification, hypoxia, and fish mortality. Eutrophication of the aquatic environment is caused by high nitrogen concentrations, which results in a loss of biodiversity and a worsening of water quality. In this study, the natural abundance of the nitrogen stable isotope (*δ*^15^N) is measured and sampled in sediment and compared with the total dissolved nitrogen in four main Chinese tributaries of the Hun River upper reach, including the Dasuhe, Beisanjia, Beikouqian, and Nanzamu tributaries. Results show that all surveyed tributaries except the Dasuhe showed a significant increase in DN. In addition, a significant positive correlation between the change ratio of farmland area and DN in river water was detected, suggesting that the increase in nitrogen in river water from 2011 to 2016 is due to agriculture. In addition, the outcomes of this study showed that government measures did change the type of nitrogen sources in watersheds. Unfortunately, because of insufficient execution and lack of environmental protection knowledge among farmers, no significant effects on nitrogen reduction in the Upper Hun River Basin were detected. As a recommendation, the government should pay more attention to the implementation process and then formulate policies, strengthen supervision, and increase farmer environmental awareness.

## Figures and Tables

**Figure 1:** Sampling locations and the WTF running status.

**Figure 2:** Changes in dissolved total nitrogen concentration and the proportion of inorganic nitrogen in the four tributaries.

**Figure 3:** Changes in sediment *δ*^15^N values in each sampling point.

**Figure 4:** Changes in mean sediment *δ*^15^N values in the four tributaries.

RETRACTED

**Figure 5:** Range of the sediment *δ*^15^N value and TN concentration in each sampling point.

**Figure 6:** Correlation analysis of the change rate of total nitrogen dissolved in river water and change rate of farmland proportion.

**Table 1:** Changes in main background information from the year 2011 to the year 2016.

Tributaries	Population density (people·km^−2^)		Farmland area percent (%)		Villages/townspercent (%)	
	2011	2016	2011	2016	2011	2016
Dasuhe	31	33	5.1	2.9	0.19	0.140771
Nankouqian	70	66	16.3	10.2	0.61	0.54912
Beisanjia	54	57	2.6	7.7	0.46	0.587495
Nanzamu	320	314	17.9	10.9	4.50	4.823265

**Table 2:** Stable nitrogen isotope values of main nitrogen sources to Hun River aquatic systems.

Type of nitrogen sources	Soil		Chemical fertilizers	Livestock manure	Wastewater
	Forest	Field			
*δ* ^15^N (%)^*∗*^	4.6 (0.4) (2.5–5.7)	5.1 (0.4) (3.6–6.22)	0.35 (0.5) (−1.84–2.8)	7.6 (1.0) (5.8–10.1)	25.5 (3.2) (18.2–38.3)
Number of samples	9	15	10	6	6

^*∗*^ Values are mean (± standard deviation) with the range between parentheses.

**Table 3:** Total nitrogen and stable nitrogen isotope values of sediment and composition of water nitrogen from 2011 to 2016.

Tributary	Station code	2011					2016				
		Sediment			Water		Sediment			Water	
		*n*	TN ± S.D. (%)	*δ* ^15^N ± S.D. (%)	Inorganic nitrogen (mg/L)	Dissolved nitrogen (mg/L)	*n*	TN ± S.D. (%)	*δ* ^15^N ± S.D. (%)	Inorganic nitrogen (mg/l)	Dissolved nitrogen (mg/l)
Dasuhe	HR1	3	0.24 (0.1)	2.2 (0.2)	1.8	1.9	3	0.04 (0.01)	4.7 (0.7)	2.8	2.8
	HR2	4	0.31 (0.1)	3.6 (0.6)	1.0	1.3	3	0.12 (0.01)	5.6 (0.3)	1.9	2.3
	HR3	3	0.23 (0.02)	4.0 (0.2)	1.7	1.8	3	0.06 (0.01)	5.9 (0.4)	2.1	2.3
	HR4	2	0.14 (0.06)	3.3 (0.1)	4.8	5.5	3	0.12 (0.01)	6.1 (0.4)	1.6	1.6
	HR5	1	0.14	4.2	0.7	0.7	3	0.13 (0.03)	5.9 (0.1)	1.7	1.7

Nankouqian	HR6	3	0.17 (0.2)	2.2 (0.1)	5.7	7.2	2	0.29 (0.01)	4.3 (0.1)	0.5	1.5
	HR7	3	0.11 (0.1)	3.5 (0.1)	2.3	2.5	3	0.04 (0.01)	7.0 (0.3)	4.2	4.2
	HR8	3	0.07 (0.02)	4.5 (0.1)	1.8	2.1	3	0.22 (0.04)	7.4 (0.2)	2.8	2.8
	HR9	3	0.09 (0.02)	5.4 (0.1)	1.9	2.0	3	0.04 (0.01)	10.4 (3.2)	4.1	4.2
	HR10	4	0.21 (0.03)	5.9 (0.2)	0.4	0.4	3	0.09 (0.01)	9.2 (1.3)	5.9	8.2

Beisanjia	HR11	3	0.17 (0.03)	3.7 (0.07)	1.4	1.8	3	0.15 (0.02)	6.6 (0.2)	4.0	5.3
	HR12	2	0.04 (0.03)	5.2 (0.1)	1.4	1.6	3	0.32 (0.02)	4.8 (0.5)	2.8	2.8
	HR13	3	0.12 (0.03)	5.8 (0.1)	0.5	0.6	3	0.46 (0.03)	3.8 (0.1)	3.3	3.3

Nanzamu	HR14	2	0.45 (0.1)	2.6 (0.1)	3.0	3.2	3	0.22 (0.01)	6.6 (0.1)	3.7	4.2
	HR15	3	0.63 (0.2)	4.2 (0.1)	2.2	2.3	3	0.27 (0.01)	6.0 (0.2)	5.2	7.3
	HR16	3	0.57 (0.1)	5.9 (0.1)	7.9	7.9	3	0.28 (0.01)	6.4 (0.2)	5.7	9.3
	HR17	4	0.34 (0.02)	9.1 (0.7)	4.6	4.8	3	0.28 (0.01)	6.0 (0.1)	5.4	5.7

Hun River stem	HS1	—	—	—	—	—	3	0.60 (0.02)	4.9 (0.2)	3.3	5.1
	HS2	—	—	—	—	—	3	0.17 (0.02)	10.1 (2.4)	3.1	3.2
	HS3	—	—	—	—	—	3	0.13 (0.02)	8.8 (0.5)	2.8	3.0
	HS4	—	—	—	—	—	3	0.04 (0.02)	6.4 (0.3)	2.9	4.3
	HS5	—	—	—	—	—	3	0.18 (0.02)	6.7 (0.4)	3.3	5.2
	HS6	—	—	—	—	—	3	0.11(0.02)	8.5 (0.7)	3.3	3.9

“—” means that this sampling point was not established in 2011.

RETRACTED

## Data Availability

The data that support the findings of this study are available from the corresponding author upon reasonable request.

## References

[1] Gruber N., Galloway J. N. (2008). An Earth-system perspective of the global nitrogen cycle. *Nature*.

[2] Zhang X., Zhang Y., Shi P., Bi Z., Shan Z., Ren L. (2021). The deep challenge of nitrate pollution in river water of China. *Science of the Total Environment*.

[3] Min J., Shi W. (2018). Nitrogen discharge pathways in vegetable production as non-point sources of pollution and measures to control it. *Science of the Total Environment*.

[4] Finkler Ferreira T., Crossetti L. O., Motta Marques D. M., Cardoso L., Fragoso C. R., van Nes E. H. (2018). The structuring role of submerged macrophytes in a large subtropical shallow lake: clear effects on water chemistry and phytoplankton structure community along a vegetated-pelagic gradient. *Limnologica*.

[5] De Girolamo A. M., Balestrini R., D’Ambrosio E., Pappagallo G., Soana E., Lo Porto A. (2017). Anthropogenic input of nitrogen and riverine export from a Mediterranean catchment. The Celone, a temporary river case study. *Agricultural Water Management*.

[6] Díaz F. J., O’Geen A. T., Dahlgren R. A. (2012). Agricultural pollutant removal by constructed wetlands: implications for water management and design. *Agricultural Water Management*.

[7] Jiang J., Li S., Hu J., Huang J. (2014). A modeling approach to evaluating the impacts of policy-induced land management practices on non-point source pollution: a case study of the Liuxi River watershed, China. *Agricultural Water Management*.

[8] Su X., Wang H., Zhang Y., Jin H. (2013). The present situation and evaluation of nitrate pollution in soil in a regional aeration zone: using the proluvial fan agriculture irrigation district of Hunhe River in northeast China as an example. *Environmental Earth Sciences*.

[9] Grizzetti B., Pretato U., Lassaletta L., Billen G., Garnier J. (2013). The contribution of food waste to global and European nitrogen pollution. *Environmental Science & Policy*.

[10] Klages S., Heidecke C., Osterburg B. Nitrogen surplus-A unified indicator for water pollution in europe?. *Water*.

[11] Smith L., Siciliano G. (2015). A Comprehensive Review of Constraints to Improved Management of Fertilizers in China and Mitigation of Diffuse Water Pollution from Agriculture. *Agriculture Ecosystems & Environment*.

RETRACTED

[12] Zhao X., Huang M. (2019). Spatial distribution of nitrogen of topsoil in the wangdonggou watershed of the loess plateau. *Research of Soil and Water Conservation*.

[13] Hu Y., Zhang K., Li Y., Sun Y., Li H., Yang G. (2021). Human activities increase the nitrogen in surface water on the eastern loess plateau. *Geofluids*.

[14] Wang R., Xu T., Yu L., Zhu J., Li X. (2013). Effects of land use types on surface water quality across an anthropogenic disturbance gradient in the upper reach of the Hun River, Northeast China. *Environmental Monitoring and Assessment*.

[15] Nadeau T. (2017). Hydrological connectivity between headwater streams and downstream waters: how science can inform policy. *Journal of the American Water Resources Association*.

[16] Yang L., Lei K. (2018). Effects of land use on the concentration and emission of nitrous oxide in nitrogen-enriched rivers. *Environmental Pollution (Amsterdam, Netherlands)*.

[17] Yang X., Liu Q., Fu G., He Y., Luo X., Zheng Z. (2016). Spatiotemporal patterns and source attribution of nitrogen load in a river basin with complex pollution sources. *Water Research*.

[18] Xu J., Jin G., Tang H. (2018). Assessing temporal variations of Ammonia Nitrogen concentrations and loads in the Huaihe River Basin in relation to policies on pollution source control. *Science of the Total Environment*.

[19] Gökkaya K., Budhathoki M., Christopher S. F., Hanrahan B. R., Tank J. L. (2017). Subsurface tile drained area detection using GIS and remote sensing in an agricultural watershed. *Ecological Engineering*.

[20] Bannon R. O., Roman C. T. (2008). Using stable isotopes to monitor anthropogenic nitrogen inputs to estuaries. *Ecological Applications*.

[21] Chibwe L., Manzano C. A., Muir D. (2019). Deposition and source identification of nitrogen heterocyclic polycyclic aromatic compounds in snow, sediment, and air samples from the athabasca oil sands region. *Environmental Science & Technology*.

[22] Kohzu A., Miyajima T., Tayasu I. (2008). Use of stable nitrogen isotope signatures of riparian macrophytes as an indicator of anthropogenic N inputs to river ecosystems. *Environmental Science & Technology*.

[23] Choi W. J., Han G. H., Lee S. M. (2007). Impact of land-use types on nitrate concentration and *δ*^15^N in unconfined groundwater in rural areas of Korea. *Agriculture, Ecosystems & Environment*.

[24] McClelland J. W., Valiela I. (1998). Linking nitrogen in estuarine producers to land-derived sources. *Limnology & Oceanography*.

[25] Wang R., Tang J., Xie Z. (2015). Occurrence and spatial distribution of organophosphate ester flame retardants and plasticizers in 40 rivers draining into the Bohai Sea, north China. *Environmental Pollution (Amsterdam, Netherlands)*.

RETRACTED

[26] Ma J., Chen X., Huang B., Shi Y., Chi G. Y., Lu C. (2015). Utilizing water characteristics and sediment nitrogen isotopic features to identify non-point nitrogen pollution sources at watershed scale in Liaoning Province, China. *Environmental Science and Pollution Research*.

[27] Knöller K., Vogt C., Haupt M., Feisthauer S., Richnow H. H. (2011). Experimental investigation of nitrogen and oxygen isotope fractionation in nitrate and nitrite during denitrification. *Biogeochemistry*.

[28] Wilkinson J. L., Hooda P. S., Swinden J., Barker J., Barton S. (2018). Spatial (bio)accumulation of pharmaceuticals, illicit drugs, plasticisers, perfluorinated compounds and metabolites in river sediment, aquatic plants and benthic organisms. *Environmental Pollution (Amsterdam, Netherlands)*.

[29] Zeng X., Xu L., Liu J., Wu Y., Yu Z. (2018). Occurrence and distribution of organophosphorus flame retardants/plasticizers and synthetic musks in sediments from source water in the Pearl River Delta, China. *Environmental Toxicology & Chemistry*.

